The article "Dinitrosopiperazine-Mediated Phosphorylated-Proteins Are Involved in Nasopharyngeal Carcinoma Metastasis" was retracted in 2020. Reason: duplicated images.

# Dinitrosopiperazine-Mediated Phosphorylated-Proteins Are Involved in Nasopharyngeal Carcinoma Metastasis

**DOI:** 10.3390/ijms151120054

**Published:** 2014-11-04

**Authors:** Gongjun Tan, Xiaowei Tang, Damao Huang, Yuejin Li, Na Liu, Zhengke Peng, Zhenlin Zhang, Chaojun Duan, Jinping Lu, Guangrong Yan, Faqing Tang

**Affiliations:** 1 Medical Research Center and Clinical Laboratory, Zhuhai Hospital of Jinan University, 79 Kangning Road, Zhuhai 519000, China; E-Mails: tgj1129@163.com (G.T.); liyuejincat@163.com (Y.L.); pengzhengke@126.com (Z.P.); fromzhenlin@foxmail.com (Z.Z.); lujinping_2006@163.com (J.L.); 2 Clinical Laboratory and Medical Research Center, Xiangya Hospital, Central South University, 87 Xiangya Road, Changsha 410008, China; E-Mails: huangdamao@hotmail.com (D.H.); liuna8542@163.com (N.L.); duancjxy@126.com (C.D.); 3 Metallurgical Science and Engineering, Central South University, 21 Lushan South Road, Changsha 410083, China; E-Mail: tangxw19907@hotmail.com; 4 Institute of Life and Health Engineering, National Engineering and Research Center for Genetic Medicine, Jinan University, 601 Huangpu Road West, Guangzhou 510632, China; E-Mail: jxygr007@126.com

**Keywords:** dinitrosopiperazine, nasopharyngeal carcinoma, metastasis, protein phosphorylation, proteomics

## Abstract

*N*,*N*'*-*dinitrosopiperazine (DNP) with organ specificity for nasopharyngeal epithelium, is involved in nasopharyngeal carcinoma (NPC) metastasis, though its mechanism is unclear. To reveal the pathogenesis of DNP-induced metastasis, immunoprecipitation was used to identify DNP-mediated phosphoproteins. DNP-mediated NPC cell line (6-10B) motility and invasion was confirmed. Twenty-six phosphoproteins were increased at least 1.5-fold following DNP exposure. Changes in the expression levels of selected phosphoproteins were verified by Western-blotting analysis. DNP treatment altered the phosphorylation of ezrin (threonine 567), vimentin (serine 55), stathmin (serine 25) and STAT3 (serine 727). Furthermore, it was shown that DNP-dependent metastasis is mediated in part through ezrin at threonine 567, as DNP-mediated metastasis was decreased when threonine 567 of ezrin was mutated. Strikingly, NPC metastatic tumors exhibited a higher expression of phosphorylated-ezrin at threonine 567 than the primary tumors. These findings provide novel insight into DNP-induced NPC metastasis and may contribute to a better understanding of the metastatic mechanisms of NPC tumors.

## 1. Introduction

Nasopharyngeal carcinoma (NPC) is more prominent in southeastern China than in western countries. Epidemiological studies have indicated that infection with Epstein–Barr virus (EBV), dietary habits, and genetic susceptibility might be critical cofactors in the development of NPC [1]. NPC is highly invasive and metastatic, and approximately 90% of patients show cervical lymph node metastasis at first diagnosis as a result of its silent, deep-seated location and non-specific symptoms [2]. In recent years, developments in diagnostic methods, radiotherapeutic techniques and chemotherapy regimens have provided significant survival benefits for patients with locally advanced NPC. Nonetheless, the survival rate with advanced NPC remains low as a result of high rates of local recurrence and distantmetastasis [3,4,5,6]. EBV participates in NPC metastasis through its encoding of virusprotein and microRNA (miR). EBV encodes various oncoproteins, including latent membrane protein 1 (LMP1), latent membrane protein 2A (LMP2A), EBV nuclear antigen 1 (EBNA1) and EBV-encoded glycoprotein (BALF1). Generally, LMP1 expression is positively associated with NPC metastasis [7]. LMP1 promotes NPC metastasis through inducing the expression of tyrosylprotein sulfotransferase-1 and tyrosine sulfation of chemokine receptor 4 [8]. LMP1 also up-regulates matrix metalloproteinase 9 (MMP9), which may be a pivotal effector of EBV-induced invasion-promotion. NF-κB-mediated transcriptional up-regulation of tumor necrosis factor α-induced protein 2 (TNFAIP2) by LMP1 promotes NPC cell motility [9]. LMP1 suppresses miR-204 expression by activating STAT3, and miR204 inhibits EBV-positive C666-1 cell invasion and metastasis partly through targeting cdc42 [10]. LMP2A, a well-known NPC activator, induces epithelial-mesenchymal transition (EMT) and has been shown to exert a promoting-effect in tumor metastasis. LMP2A could induce EMT by activating MTA1 at the translational level via activating the mTOR signaling and the 4EBP1-eIF4E axis [11]. LMP2A also promotes NPC cell invasion through ERK/Fra-1-mediated induction of MMP9 [12]. EBV nuclear antigen 1 (EBNA1) induces NPC cell EMT [13], and BALF1 facilitates tumor formation and metastasis potential [14]. Additionally, EBV-encoded miR-BART9 promotes tumor metastasis by targeting E-cadherin in NPC [15]. However, the highly metastatic mechanism has not been clarified. Our previous study showed that exposure to *N,N*'-dinitrosopiperazine (DNP) is associated with NPC metastasis, and that DNP can promote tumor metastasis [16,17,18,19]. However, the underlying mechanism responsible for induction and promotion of NPC metastasis by DNP remains unknown.

The article "Dinitrosopiperazine-Mediated Phosphorylated-Proteins Are Involved in Nasopharyngeal Carcinoma Metastasis" was retracted in 2020. Reason: duplicated images.

Protein phosphorylation is a central mechanism by which cells orchestrate regulatory and signaling processes. Phosphorylation can regulate a variety of important protein functions, including subcellular localization, protein degradation and stabilization, as well as biochemical activities [20,21]. Protein phosphorylation and dephosphorylation are regulated by a careful balance of the competing activities of protein kinases and protein phosphatases. In the development of cancer, carcinogens may cause constitutive activation of some protein kinases such as Rho-kinase, protein kinase (PKC), epidermal growth factor (EGFR), breakpoint cluster region-Abelson fusion (BCR-Abl) and receptor tyrosine kinase ErbB-2 [22,23,24]. The hyper activation of some protein kinases is also associated with tumor progression to metastatic phenotypes [25].

As a carcinogen for NPC, DNP may also induce phosphorylated-protein expression, and mediate multi-signal pathways involved in NPC metastasis. To fully understand the DNP-mediated signaling pathways and identify novel signaling components, we here employed proteomics technology to comprehensively identify the DNP-regulated phosphoproteins and phosphosites by using high resolution mass spectrometry (MS). Twenty-six phosphoproteins were found to be regulated by DNP, most of which were not previously reported to be involved in NPC metastasis. Analysis of this vast information helps us better understand the complex regulatory mechanisms of DNP regulating NPC metastasis.

## 2. Results

### 2.1. Identification of Non-Cytotoxic Concentrations of DNP in 6-10B NPC Cells

DNP is an important carcinogenic *N*-nitroso compound for NPC, and its chemical structure is shown in Figure 1A. In the present study, we determined the non-cytotoxic concentration of DNP by treating 6-10B cells with various DNP concentrations for 24 or 48 h. Cell viability was estimated by measurement of lactate dehydrogenase (LDH) activity in the cell culture media following DNP treatment. Compared with the control, LDH activity was not significantly altered after 24 h at 2–10 μM DNP, nor was there a difference when DNP treatment was extended to 48 h (Figure 1B; *, *p* < 0.05). As a result, this concentration range was used in all subsequent experiments.

**Figure 1:** Non-cytotoxic concentration of *N*,*N*'-dinitrosopiperazine (DNP) in 6-10B cells. (**A**) Structure of DNP, an *N*-nitroso compound; (**B**) 6-10B cells were treated with 2, 4, 6, 8, 10, 15, 20, 40, or 60 μM DNP for 48 h, and then LDH activity in the cell culture media were detected. Data are presented as means ± S.D. from three independent experiments, statistically analyzed using the Student’s *t*-test (*, *p* < 0.05).

### 2.2. DNP Induces the Invasion and Motility of 6-10B Cells

6-10B cells have a low metastasis, and so was used to determine whether DNP induces NPC cell metastasis. To determine whether DNP can induce invasion and motility, Matrigel-coated Boyden chambers were used to measure cell invasion, and uncoated Boyden chambers were used for assessment of cell motility. After DNP treatment, the number of invading cells dramatically increased in both the Matrigel-coated Boyden chamber (Figure 2A-b) and the uncoated Boyden chamber (Figure 2A-d) compared to the controls (Figure 2A-a,c). This result indicates that DNP treatment induced an increase in the invasion and motility of 6-10B cells. In dose-course experiments, 6-10B cells were treated with 0, 1, 2, 4 or 6 μM DNP for 24 h and seeded into Boyden chambers, and cells that invaded the lower chamber were counted. The number of invading cells significantly increased after DNP treatment in a dose-dependent manner (Figure 2B, lanes 2 to 5 *vs.* lane 1; *, *p* < 0.05). At 6 μM DNP, the increase in invasion was 321.7% (Figure 2B, lane 5). A similar effect was observed on the motility of DNP-treated cells (Figure 2C, lanes 2 to 5 *vs.* lane 1; *, *p* < 0.05). Cell motility increased by 455.2% after treatment with 6 μM DNP (Figure 2C, lane 5). These results indicate that DNP can induce NPC cell motility and invasion.

The article "Dinitrosopiperazine-Mediated Phosphorylated-Proteins Are Involved in Nasopharyngeal Carcinoma Metastasis" was retracted in 2020. Reason: duplicated images.

**Figure 2:** DNP-mediated NPC cell motility and invasion. To determine DNP-induced invasion and motility, Boyden chambers coated with Matrigel were used to measure 6-10B cell invasion, and those uncoated with Matrigel were used for cell motility. The cells invading the lower surface of the membrane were fixed with methanol and stained with hematoxylin and eosin. (**Aa**) 6-10B treated with 0.01% DMSO–PBS in Boyden chamber with coated Matrigel; (**Ab**) 6-10B cells treated with DNP 4 μM in Matrigel-coated Boyden chamber; Scale bar (a,b), 5 μm; (**Ac**) 6-10B treated with 0.01% DMSO–PBS in uncoated with Matrigel; (**Ad**) 6-10B cells with DNP treatment in uncoated with Matrigel. Scale bar (c,d), 10 μm. Arrows, invaded cell. In concentration-course assays, 6-10B cells were treated with 0, 1, 2, 4, 6 μM DNP for 24 h. Treated cells were subjected to analyses for motility and invasion. Random fields were counted for invading cells under a light microscope; (**B**) invasion of 6-10B cells at various concentrations; (**C**) motility of 6-10B cells at various concentrations. Results were statistically analyzed by one-way analysis of variance (ANOVA) with *post-hoc* Dunnett’s test (*, *p* < 0.05).

### 2.3. Proteomic Analysis of DNP-Mediated Phosphoprotein Expression

Proteomic analysis was performed on immunoprecipitated proteins using antibodies against phosphoserine and phosphothreonine epitopes. Following immunoprecipitation, phosphoproteins were separated by high-resolution two-dimensional difference gel electrophoresis (2D-DIGE). Well-resolved and reproducible 2D-DIGE patterns of proteins on a clear background were attained in the immunoprecipitates of the control (Figure 3a) and DNP-treated cells (Figure 3b) using the phosphoserine antibody. More than 100 protein spots were detected on the two-dimensional electrophoresis gels and localized in the isoelectric point (*p*I) range of *p*I 3–10 with relative molecular masses of 10–200 kDa. Similarly, more than 100 protein spots were detected in immunoprecipitates of the control (Figure 3c) and DNP-treated cells (Figure 3d) using the phosphothreonine antibody, with a similar range of *p*I and molecular masses as above. Using image Master 2-DE Elite 4.01 (Pierce, Rockford, IL, USA), we found that the separation was clear in the lower molecular weight range toward the acidic pH. Horizontal streaks were apparent for proteins in the higher molecular range. The experiment was repeated three times, and three silver-stained 2-DE profiles of each sample were in accordance. A total of 60 resolved and matched spots were chosen randomly to calculate the deviation of the spot position. The spot position deviation was 0.7987 ± 0.216 mm in the IEF direction and 1.297 ± 0.317 mm in the SDS-PAGE direction. These two-dimensional proteins were quantified and compared with the control, there were 26 highly expressed protein spots (>1.5-folds) in the DNP-treated cells. One protein-free parallel gel piece served as a negative control. The gel spots were destained in the destaining solution. The samples were analyzed with an Applied Biosystems Voyager System 4307 MALDI-TOF Mass Spectrometer (Thermo Electron, Bremen, Germany). A trypsin-fragment peak served as an internal standard for mass calibration. Proteins were identified with peptide mass fingerprinting data by searching software PeptIdent [26], and the searching parameters were set (for details please see Materials and Methods Section). The results are summarized in Table 1.

The article "Dinitrosopiperazine-Mediated Phosphorylated-Proteins Are Involved in Nasopharyngeal Carcinoma Metastasis" was retracted in 2020. Reason: duplicated images.

**Figure 3:** Proteomic analysis of phosphoproteins mediated by DNP. The total proteins in 6-10B cells with or without DNP treatment were extracted, and the phosphoproteins were immunoprecipitated (IPed) using a phosphoserine-antibody or phosphothreonine-antibody respectively. The IPed proteins were then separated on an IPG strip (pH 3-10L, 180 mm × 3 mm × 0.5 mm) on IPG phor (Amersham Biosciences, Piscataway, NJ, USA) and were run through a 9%–16% SDS-PAGE (Bio-Rad, Hercules, CA, USA) as per the manufacturer’s instructions. After electrophoresis separation, the protein spots were visualized by silver-based staining technique with the protein silver stain kit (Amersham Biosciences). (**a**) IP protein with serine-antibody in 6-10B cells treated with 0.01% DMSO; (**b**) IP protein with serine-antibody in 6-10B cells treated with 4 μM DNP; (**c**) IP protein with threonine-antibody in 6-10B cells treated with 0.01% DMSO; (**d**) IP protein with threonine-antibody in 6-10B cells treated with 4 μM DNP. Three independent experiments were carried out and representative figures are shown. Arrows: the highlyexpressed proteins.

### 2.4. Validation of Differential Phosphoproteins

To further verify that the proteomically identified phosphoproteins were regulated by DNP, highly expressed markers, ezrin, vimentin, stathmin and STAT3 were respectively detected using phospho-antibody by Western-blotting. Compared with the control, phospho-ezrin Thr567 (Figure 4A), phospho-vimentin Ser55 (Figure 4B), phospho-stathmin Ser25 (Figure 4C) and phospho-STAT3 Ser727 (Figure 4D) were increased in 6-10B cells following DNP treatment. The changing trends of the Western-blotting results for all the selected proteins were consistent with the proteomic data. DNP treatment increases the expression of phospho-ezrin, phospho-vimentin, phospho-stathmin and phospho-STAT3.

**Table 1:** Identification of differential phosphoproteins in DNP-treated NPC cells by 2D-DIGE and MS.

No.	Protein Name	Uniprot Accession	*M*_r_	*p*I
1	Heat shock cognate 71 kDa protein	P11142	71,082	5.31
2	Keratin,type II cytoskeletal 8	P05787	53,669	5.57
3	TUBB protein	P07437	50,097	4.88
4	Vimentin	P08670	53,679	5.16
5	Heterogeneous nuclear ribonucleoprotein k	P61978	51,233	5.22
6	60 kDa Heat shock protein	P10809	61,191	5.66
7	Keratin type II cytoskeletal 8	P05787	53,669	5.54
8	Laminin receptor 1	P08865	32,951	4.88
9	Creatine kinase B-type	P12277	42,911	5.24
10	ATP synthase D chain mitochondrial	O75947	18,541	5.22
11	Ezrin	P003370	69,282	5.36
12	Keratin,type II cytoskeletal 18	P05783	48,031	5.34
13	Nucleoside diphosphate kinase A	P15531	17,311	5.79
14	Heat shock protein β-1	P04792	22,831	5.87
15	Glutathione *S*-transferase P1	P09211	23,572	5.49
16	Protein DJ-1	Q99497	19,889	6.38
17	3-Hydroxyisobutyrate dehydrogenase mitochondrial precursor (3HIDH)	P31937	35,711	8.29
18	Stathmin	P16949	17,199	5.81
19	Annexin A3	P12429	36,524	5.67
20	Basic transcription factor 3	P20071	17,688	6.77
21	Ribosomal protein P2	P56671	11,658	4.32
22	Putative NF-κB-activating protein	Q34578	26,097	8.51
23	Microtubule-associated serine	P48618	98,398	5.67
24	c-Myc-responsive protein	O43598	19,321	5.05
25	Growth factor receptor-bound protein 2	P62993	25,209	5.71
26	Proliferating cell nuclear antigen	P12004	29,097	4.61

### 2.5. DNP-Mediated Invasion and Motility Is Phospho-Ezrin Thr567 Dependent

Ezrin, vimentin, stathmin and STAT3 are all associated with cancer metastasis, and they have each been shown to promote tumor cell migration and invasion [27,28,29,30]. To elucidate whether DNP-mediated phosphoproteins are directly involved in NPC metastasis, we chose to further investigate ezrin. We transfected 6-10B cells with low levels of ezrin and metastatic potential with pcDNA3.1-ezrin. After DNP treatment, ezrin and phosphor-ezrin expression were increased (Figure 5A), and its invasion and motility were also dramatically increased after being transfected (Figure 5B, lane 1 *vs.* 5; Figure 5C, lane 1 *vs.* 5; *, *p* < 0.05). The cells were then transfected using pcDNA3.1-ezrin-mutant, in which the ezrin phosphorylation site Thr567 was mutated, and the expression of phospho-ezrin Thr 567 did not increase (Figure 5A), and neither the invasion nor the motility were increased after DNP treatment (Figure 5B, lane 4; Figure 5C, lane 4). However, DNP could effectively induce cell invasion (Figure 5B, lane 5 *vs.* 6, *p* < 0.05) and motility (Figure 5C, lane 5 *vs.* 6, *p* < 0.05) when the ezrin phosphorylation site Thr567 was not mutated. These results indicate that DNP mediates phosphorylated-ezrin expression, and thereby increases the cell invasion and motility involved in NPC metastasis.

The article "Dinitrosopiperazine-Mediated Phosphorylated-Proteins Are Involved in Nasopharyngeal Carcinoma Metastasis" was retracted in 2020. Reason: duplicated images.

**Figure 4:** Validation of the representative phosphoproteins by Western-blotting. Representative proteins ezrin (**A**); vimentin (**B**); stathmin (**C**); STAT3 (**D**) of the immunoprecipitated proteins were detected by Western-blotting using anti-serine or threonine phosphorylation antibody. IgG served as the control. The relative Western-blotting ratio of phosphorylation levels of every protein was normalized to its corresponding proteomic data.

**Figure 5:** DNP induces motility and invasion through ezrin phosphorylation. (**A**) 6-10B cells were transfected using pcDNA3.1, pcDNA3.1-ezrin or the pcDNA3.1-ezrin mutant. Ezrin and phospho-ezrin were detected with Western-blotting analysis; the invasion (**B**) and motility (**C**) were detected in 6-10B-mock, 6-10B-ezrin and 6-10B-ezrin mutant cells with or without DNP treatment. Data are presented as means ± SD from three independent experiments. Results were analyzed by one-way ANOVA with *post-hoc* Dunnett’s test (*, *p* < 0.05).

### 2.6. Expression of Phospho-Ezrin Thr567 in Metastatic NPC

To further determine whether DNP-mediated ezrin phosphorylation at Thr567 is associated with NPC metastasis *in vivo*, phospho-ezrin Thr567 was detected in 27 cases of primary NPC tumors and 21 NPC metastatic nodes using immunohistochemistry. The results showed that the positive rate of phospho-ezrin was 80.95% (17/21) in metastatic nodes, while 40.74% (11/27) in primary tumors. The expression of phospho-ezrin Thr567 was higher in the metastatic tumors (Figure 6, panel f) than in primary tumors (Figure 6, panel e).

The article "Dinitrosopiperazine-Mediated Phosphorylated-Proteins Are Involved in Nasopharyngeal Carcinoma Metastasis" was retracted in 2020. Reason: duplicated images.

**Figure 6:** Phospho-ezrin and ezrin expression in NPC metastatic nodes. Phospho-ezrin and ezrin were detected in the primary and metastatic NPC samples using immunohistochemistry. (**a**,**b**) primary NPC and metastatic tumor sections were stained with hematoxylin and eosin; (**c**,**d**) stained with antibodies against ezrin; (**e**,**f**) stained with phospho-ezrin at Thr567; (**g**,**h**) stained with IgG, served as a blank control. Arrow, positive cells. Original magnification, ×400. Scale bar, 5 μm. H&E, hematoxylin and eosin.

## 3. Discussion

As a specific carcinogen for NPC [16,17], DNP is likely involved NPC metastasis [19], but its mechanism is not clear. At first, we confirmed DNP-mediated NPC cell metastasis, and found that DNP exactly induced NPC cell motility and invasion. These findings suggest that DNP may activate some signal pathways when DNP mediates NPC metastasis. In the present work, phosphoprotein proteomics was used to comprehensively identify DNP-regulated phosphoproteins. We found that DNP increased the expression levels of 26 phosphoproteins, including ezrin, vimentin, stathmin and STAT3, which are associated with cellular growth, proliferation, cell motility, and invasion signaling pathways.

Western-blotting analysis was used to confirm the effect of DNP on a subset of phosphoproteins. Our results showed that DNP induces the expression of phospho-ezrin, phospho-vimentin, phospho-stathmin and phospho-STAT3 at specific epitopes. To elucidate further the involvement of phosphoprotein signaling in DNP-induced NPC metastasis, we examined the requirement for ezrin Thr567 phosphorylation. Ezrin is associated with tumor metastasis [31,32,33,34], including NPC [34]. Ezrin may control multiple pathways and promote tumor metastasis [35]. Our previous study has verified that DNP induces ezrin phosphorylation at Thr567, and increases the motility and invasion of cells, and promotes tumor metastasis [18]. To further confirm this hypothesis, we used 6-10B cells with low baseline ezrin expression, and transfected this cell line with ezrin or mutated ezrin (Thr567 mutated to Ala567), and observed the effects of DNP on cell motility and invasion. Interestingly, DNP induced cell motility and invasion in cells transfected with ezrin, but did not induce these effects in cells transfected with the ezrin mutant. As a cytoskeleton organizer, ezrin is involved in various cellular functions such as cell adhesion, migration, and the organization of cell surface structures [36,37]. Phosphorylation at a conserved threonine residue in the *C* terminus (Thr567) is acritical mechanism for regulating the function of ezrin [38], including its important role in cell metastasis. The induction of ezrin phosphorylation at Thr567 by DNP may therefore be involved in the metastasis of NPC cells.

The article "Dinitrosopiperazine-Mediated Phosphorylated-Proteins Are Involved in Nasopharyngeal Carcinoma Metastasis" was retracted in 2020. Reason: duplicated images.

Vimentin is the major intermediate filament protein of mesenchymal cell. It emerges as an organizer of a number of critical proteins involved in attachment, migration, and cell signaling [28]. Vimentin is over-expressed in various epithelial cancers, and its over-expression correlates well with accelerated tumor growth, invasion, and poor prognosis [29]. Vimentin has also been recognized as a marker for EMT, wherein epithelial cells loosen cell–cell adhesion structures and become migratory [30]. They modulate their polarity, cytoskeleton organization, increase expression of vimentin filaments and down-regulate cytokeratins. They become isolated, mobile and resistant to anoikis [39], enabling normally sessile epithelial tumor cells to move away from the primary tumor and metastasize. The highly dynamic and complex phosphorylation of vimentin seems to be a likely regulator mechanism for these functions [28]. Stathmin is another important protein which destabilizes microtubules. The essential function of stathmin is closely associated with its phosphorylation status. Stathmin is overexpressed in many human cancers and has a significant relationship with clinical characteristics such as grade, tumor size and prognosis [40]. DNP may also mediate NPC metastasis through inducing phosphorylation of stathmin Ser25. STAT3 is one of six members of a family of transcription factors [41] that has previously been associated with inflammation, cellular transformation, survival, proliferation, invasion, angiogenesis, and metastasis of cancer. Various types of carcinogens, radiation, viruses, growth factors, oncogenes, and inflammatory cytokines are known to activate STAT3. Phosphorylation of STAT3 leads to its dimerization, nuclear translocation, DNA binding, and downstream gene transcription [42]. Based on these findings, we speculate that DNP may also mediate NPC metastasis through inducing phosphorylation of vimentin Ser25, stathmin Ser25 and STAT3 Ser727, a possibility that needs further investigation.

Taken together, the results presented here demonstrate a positive correlation between DNP exposure and phosphorylation of proteins including ezrin, vimentin, stathmin and STAT3. The interplay between DNP and protein phosphorylation provides a potential mechanistic explanation for a metastasis mechanism in NPC cells, and may provide a new therapeutic strategy for NPC patients.

The article "Dinitrosopiperazine-Mediated Phosphorylated-Proteins Are Involved in Nasopharyngeal Carcinoma Metastasis" was retracted in 2020. Reason: duplicated images.

## 4. Materials and Methods

### 4.1. Reagents and Antibodies

DNP was a kind gift from the Cancer Research Institute of Central South University (Changsha, China), and its chemical structure is shown in Figure 1A. Chemical reagents, including Tris, HCl, sodium dodecyl sulfate (SDS), Na_2_S_2_O_3_, K_3_Fe(CN)_6_, TPCK-trypsin, NH_4_HCO_3_, acrylamide, urea, thiourea, NP-40, Triton X-100, dl-dithiothreitol (DTT), phenylmethane-sulfonyl-fluoride (PMSF), CHAPS, dimethyl sulfoxide (DMSO), and pharmolyte were purchased from Sigma–Aldrich (St. Louis, MO, USA). Antibodies against ezrin, vimentin, stathmin, STAT3 and their phosphoepitopes (ezrin Thr567, vimentin Ser55, STAT3 Ser727), and the antibodies against phosphoserine and phosphothreonine were all purchased from Cell Signaling Technology (Danvers, MA, USA). The secondary antibodies, horseradish peroxidase-linked anti-mouse immunoglobulin G and anti-rabbit immunoglobulin G were purchased from Santa Cruz Biotechnology, Inc. (Santa Cruz, CA, USA). Western-blotting detection regents, Glutathione-Sepharose 4B, Quikchange II site-directed mutagenesis Kit, and BCA Protein Assay kit were purchased from Amersham Biosciences (Piscataway, NJ, USA).

### 4.2. LDH Activity Assay

To detect the non-cytotoxic concentration of DNP to 6-10B cells, the LDH activity in cell culture media was detected after DNP treatment. Briefly, the cells were seeded in 6-well plates at a density of 2 × 10^4^ cells/well and respectively treated with 0–50 μM DNP for 24 or 48 h at 37 °C. After the exposure period, media were collected for measurement of LDH activity using the LDH assay kit (AutecDiagnostica, Freiberg, Germany).

### 4.3. Cell Motility and Invasion Assay

For cell invasion assay, 6-10B cells were treated with the indicated concentrations of DNP for the indicated time. After DNP treatment, cells were removed by trypsinization, and their invasiveness was tested by the Boden chamber invasion assay [43]. Matrigel (Collaborative Biomedical products, Bedford, MA, USA) was diluted to 0.5 mg/L with cold filtered distilled water and applied to 8 mm pore size polycarbonate membrane filters. Treated cells were seeded to Boden chambers (Neuro Probe, Cabin John, MD, USA) at the upper part at a density of 1.5 × 10^4^ cells/well in 50 μL of serum-free-medium and then incubated for 12 h at 37 °C. The bottom chamber also contained standard medium with 20% fetal bovine serum (FBS). The cells that invaded to the lower surface of the membrane were fixed with methanol and stained with hematoxylin and eosin. Random fields were counted for invading cells under a light microscope.

To determine cell motility, cells were seeded into Boyden champers on membrane filters, which were not coated with Matrigel. Migration of cells was measured as described previously for the motility assay [43]. Statistical analysis was corrected with cell viability to clarify the effect of DNP.

The article "Dinitrosopiperazine-Mediated Phosphorylated-Proteins Are Involved in Nasopharyngeal Carcinoma Metastasis" was retracted in 2020. Reason: duplicated images.

### 4.4. Cell Culture and DNP Treatment

The human NPC cell line 6-10B with a low metastatic ability [34], was purchased from the Cancer Research Center of Sun Yatsen University (Guangzhou, China), and cells were grown in Dulbecco’s modified Eagle medium (DMEM). At about 30% confluence, the cells were treated with 4 μΜ DNP for 48 h according to the previous report [18], the control cells were treated with only 0.01% DMSO. Cell extracts were prepared as described previously [44]. Briefly, the cells were then harvested and suspended with lysis buffer (50 mM Tris–HCl pH 8.0, 1 mM EDTA, 2% SDS, 1 mM DTT, 10 mM PMSF, 1 mM NaF, 1 mM Na_3_VO_4_, and protease inhibitor cocktail). The lysate was centrifuged at 13,200 rpm at 4 °C for 30 min. The supernatant fractions were collected and protein concentrations were determined by the BCA assay (Pierce, Rockford, IL, USA).

### 4.5. Immunoprecipitation

For immunoprecipitation, 200 mg of supernatant protein was mixed with protein-G beads, incubated for 2 h, and centrifuged for 2 min at 2000 rpm for pre-clearing. Then the supernatant was incubated overnight with anti-phosphoserine or anti-phosphothreonine antibody (Cell Signaling Technology) and protein-G beads. The immunoprecipitates were collected and washed three times with RIPA buffer (50 mM Tris, pH 7.4, 150 mM NaCl, 1% NP-40, 0.25% sodium deoxycholate, 1 mM Na_3_VO_4_, 1 mM NaF and protease inhibitors) and finally subjected to proteomics analysis [45].

### 4.6. Proteomics Analysis

IPG-2D PAGE consisted of IEF that was performed (0.5 mm) on IPG phor using IPG strip (pH 3-10L, 180 mm × 3 mm × 0.5 mm) second-dimension SDS-PAGE analysis as described by the manufacturer. After electrophoresis separating, the protein spots were visualized by a silver-based staining technique with the protein silver stain kit (Amersham Biosciences, Shanghai, China). The stained 2-DE gels were scanned with Labscan software (Amersham Biosciences, Minneapolis, MN, USA) on an imagescanner. Spot intensity detection, background abstraction matching, 1-D calibration and establishment of average-gel were performed with Image Master 2-D Elite 4.01 analysis software (Pierce, Rockford, IL, USA). Protein staining of individual spots was quantified by calculation of spot volume after normalization of the image using the total spot volume normalization method. The reproducibility of spot position was calculated according to Gorbett’s method statistical analysis, which was carried out with SPSS version 10.0 (IBM, Chicago, IL, USA) and Excel [46].

The article "Dinitrosopiperazine-Mediated Phosphorylated-Proteins Are Involved in Nasopharyngeal Carcinoma Metastasis" was retracted in 2020. Reason: duplicated images.

### 4.7. Matrix-Assisted Laser Desorption/Ionization Time of Flight Mass Spectrometry (MALDI-TOF-MS)

A total of 27 highly expressed spots were excised from prepared gels using biopsy punches and transferred to a 1.5 mL siliconized eppendorf tube. One protein-free gel was treated in parallel as a negative control. The proteins in the gel were digested as previously described. The gel spots were destained in a destaining solution consisting of 100 mM Na_2_S_2_O_3_ and 30 mM K_3_Fe(CN)_6_ (1:1). The protein-containing gel spots were reduced in the reduction buffer consisted of 100 mmol/L NH_4_HCO_3_, 10 mM DTT for 1 h at 57 °C, and alkylated in the alkylation buffer consisting of 100 mM NH_4_HCO_3_ and 55 mM iodoacetamide in the dark for 30 min at room temperature. The gel pieces were dried in a vacant centrifuge. The dried gel pieces were incubated in the digestion solution consisting of 50 mM NH_4_HCO_3_, 5 mM CaCl_2_ and 0.1 g/L TPCK-trypsin for 24 h at 37 °C. The tryptic peptide mixtures were extracted and purified with a Millipore ZIPTIP TMC18 column. The purified tryptic peptide mixtures were mixed with the CCA matrix solution and vortexed lightly [47]. A volume containing CCA matrix was loaded on a stainless steel plate, and dried in the air. The samples were analyzed with an Applied Biosystems Voyager System 4307 MALDI-TOF mass spectrometer (Thermo Electron, San Jose, CA, USA).

### 4.8. Spectrometer

The spectrometer parameters were set up as following position ion reflector mode, acceleratory voltage 20 kV grid voltage 63.5% mirror voltage ratio 1, 12, N2 laser wave length 337 nm pulse width 3 ns, number of laser shots 50, acquisitive mass range 10-3 Torr. A 1000–3000 Da, and delay 100 ns, and vacuum degree 9 trypsin-fragment peak served as the internal standard for mass calibration. A list of the corrected mass peaks was the peptide mass fingerprint (PMF).

### 4.9. Database Analysis

Proteins were identified with peptide mass fingerprint data by searching software PeptIdent [26]. The search parameters were set up as 0.5 Dalton; the number of missed cleavage following: the mass tolerance was sites was allowed up to 1; and the system residue was 4; species was selected as HOMO SAPIENS (HUMAN). The peptide ion was [M + H]^+^; the isotope masses was 0.5 pH unit used; the searching range was within the experimental *p*I value and experimental *M*_r_ 20%.

### 4.10. Western-Blotting Analysis

Western-blotting was performed as described previously [45]. Briefly, 40 μg of the immunoprecipitates was separated by 10% or 12% PAGE and transferred onto a nitrocellulose membrane. The blots were subsequently incubated with 5% non-fat milk in phosphate buffer saline (PBS) for 1 h to block non-specific binding, and incubated with ezrin, vimentin, stathmin or STAT3 antibody (Biocompare, San Francisco, CA, USA) for 2 h, and then with an appropriate peroxidase-conjugated secondary antibody for 1 h. All incubations were carried out at 37 °C, and intensive PBS washing was performed after each incubation. After PBS washing, the signal was developed by 4-chloro-1-napthol/3,3'-*O*-diaminobenzidine, and relative photographic density was quantitated by a gel documentation and analysis system. IgG was used as an internal control to verify the basal level of expression and equal protein loading. Abundance ratio to β-actin was counted.

The article "Dinitrosopiperazine-Mediated Phosphorylated-Proteins Are Involved in Nasopharyngeal Carcinoma Metastasis" was retracted in 2020. Reason: duplicated images.

### 4.11. Construction of Expression Vectors and Gene Transfection

Ezrin DNA fragments were generated by polymerase chain reaction (PCR) and cloned into the BamHI/XhoIsites of the pcDNA3.1 vector (AmershamBiosciences, Shanghai, China) to generate pcDNA3.1-ezrin plasmids. The pcDNA3.1-ezrin mutant was generated using the QuikChange II Site-Directed Mutagenesis Kit [45]. 6-10B cells were transfected with pcDNA3.1 (mock), pcDNA3.1-ezrin, or the pcDNA3.1-ezrin mutant using Lipofectamine 2000 reagent (Life technologies, Inc., Shanghai, China) following the manufacturer’s suggested protocol. To confirm whether DNP promotes metastasis through ezrin phosphorylation, the transfected cells were treated with DNP, and their motility and invasiveness was quantified using the *in vitro* Boyden chamber invasion assay.

### 4.12. Immunohistochemistry

A total of 27 cases of primary NPC tumors, and 21 NPC metastatic nodes were used in this experiment. These tumors were embedded, 4 μm-thick tissue sections were cut, and deparaffinized in xylene, rehydrated in a graded alcohol series, and treated with an antigen retrieval solution (10 mM/L sodium citrate buffer, pH 6.0). The sections were incubated with anti-ezrin antibody (dilution 1:100) or phospho-ezrin antibody (dilution 1:50) overnight at 4 °C. Subsequently, the sections were incubated with a biotinylated secondary antibody (Zhongshan Company, Guangdong, China), followed by incubation with an avidin–biotin complex (Zhongshan Company, Guangdong, China) according to the manufacturer’s instructions. Finally, the tissue sections were incubated with 3',3'-diaminobenzidine (DAB) (Sigma–Aldrich) and hydrogen peroxide for 2 min, and counterstained with hematoxylin for 30 s. In negative controls, the primary antibodies were replaced with normal IgG. At least 10 high-power fields were chosen randomly, and >100 cells were counted for each section.

The article "Dinitrosopiperazine-Mediated Phosphorylated-Proteins Are Involved in Nasopharyngeal Carcinoma Metastasis" was retracted in 2020. Reason: duplicated images.

## 5. Conclusions

During DNP-mediated NPC metastasis, DNP regulates signaling pathways linked to cellular movement, and cellular growth and proliferation. DNP is involved in metastasis mainly through regulating ezrin, vimentin, stathmin, and STAT3, though the exact signal-pathways of DNP-mediated ezrin, vimentin, stathmin and STAT3 phosphorylation are not fully clear. The results here provide insights into the complexity and dynamics of DNP-mediated metastasis, and may help achieve a better understanding of the mechanisms involved in the high levels of metastatic activity in NPC.

## Abbreviations

DNP: *N*,*N*'-dinitrosopiperazine
NPC: nasopharyngeal carcinoma
MS: mass spectrometry
DTT: dl-dithiothreitol
PMSF: phenylmethane-sulfonyl-fluoride
phospho: phosphorylation
Thr: threonine
Ser: Serine
LDH: lactate dehydrogenase
PBS: phosphate-buffered saline
FBS: fetal bovine serum
DMEM: Dulbecco’s modified Eagle medium
EDTA: ethylenediaminetetraacetic acid
SDS: Sodium dodecyl sulfate
PKC: protein kinase C
EGFR: epithelial growth factor receptor
SDS-PAGE: Sodium dodecyl sulfate-polyacrylamide gel electrophoresis
IPG: immobilized pH gradient
IEF: isoelectric focusing
PMF: peptide mass fingerprint
PCR: polymerase chain reaction
EMT: epithelial-mesenchymal transition
